The article "Expression Profile and Prognostic Values of CDH Family Members in Lung Adenocarcinoma" was retracted in 2023. Reasons: signs of a paper mill; suspected computer-generated content; unreliable results or conclusions; concerns about the data.

# Expression Profile and Prognostic Values of CDH Family Members in Lung Adenocarcinoma

**DOI:** 10.1155/2022/9644466

**Published:** 2022-02-11

**Authors:** Feng Li, Bin Wan, Xiao-qing Li

**Affiliations:** ^1^Department of Oncology, The Chongqing Hospital of Traditional Chinese Medicine, Jiangbei District, Chongqing, China; ^2^Physical Examination Center, The Chongqing Hospital of Traditional Chinese Medicine, Jiangbei District, Chongqing, China

## Abstract

Many studies have confirmed that the classical cadherin (CDH) gene family may be involved in the development and progression of various tumors. However, the comprehensive assays of CDH family members in lung adenocarcinoma (LUAD) were rarely reported. In this study, our group analyzed TCGA datasets and identified 18 dysregulated CDH members in LUAD specimens. Several CDH members exhibited an increased level in LUAD specimens, such as CDH1, CDH2, CDH3, CDH4, CDH5, CDH15, CDH16, CDH17, CDH18, CDH24, and CDH26. However, some others exhibited decreased levels in LUAD specimens. Correlation analysis revealed that most CDH members were negatively regulated by the methylation of CDH genes, leading to their low expression in LUAD tissues. Survival assays identified 16 survival-related CDH members in LUAD patients. More importantly, we further performed multivariate analysis to determine the prognostic value of the above CDH family members and found that the expression levels of CDH17, CDH19, and CDH24 were an independent prognostic biomarker of the LUAD outcome. Finally, the results of functional enrichments revealed that CDH members participated in several tumor-related pathways. Collectively, our findings suggest that CDH Family members functioned as oncogenes or antioncogenes in LUAD and may be a potential biomarker for this malignancy.

## 1. Introduction

Lung cancer is a commonly diagnosed and highly aggressive tumor worldwide [1]. In China, there are no declining trends for incidence and mortality rates from 2010 to 2020 [2]. Based on histologic types and outcomes, lung adenocarcinoma (LUAD) accounts for >45% of all types of lung cancer and exhibits an increased trend in young adults and women [3]. Despite that distinct progresses have been made in the diagnostic methods and clinical treatments of LUAD, it is still a killer targeting human health with unfavorable outcomes [4, 5]. When the obvious clinical symptoms were observed in LUAD patients, they usually realize advanced stages and many patients exhibit a distant metastasis. Thus, it is very important to identify sensitive biomarkers for early screening of LUAD patients for the improvement of clinical outcomes for patients.

Classical cadherins (CDH) play a leading role in tissue morphogenesis and are involved in the regulation of adhesive interactions which are important for the formation of complex tissue architectures [6]. In recent years, more and more studies have demonstrated that they are involved in many complex processes, such as angiogenesis, morphogenesis, cellular communication, cellular signaling, cellular recognition, and neurotransmission [7, 8]. The function of controlling cellular adhesion and binding with other cells and ECM made it play an important part for cell differentiation, growth, and migration [9]. In recent years, more and more studies have reported the frequent dysregulation of CDH family members in many types of tumors and several of them have been functionally clarified in several tumors [10, 11]. For instance, CDH4 expression levels were distinctly increased in osteosarcoma and its silence suppressed the proliferation and invasion of osteosarcoma cells [12]. CDH12 expression was found to be distinctly upregulated in colorectal cancer, and its silence exhibited a suppressor function on the abilities of the proliferation and metastasis of colorectal cancer cells [13]. The findings highlighted the important roles of CDH family members in the progression of various tumors. In this study, we aimed to explore the expressing pattern and clinical significance of CDH family members in LUAD using bioinformatics analysis based on TCGA datasets.

The article "Expression Profile and Prognostic Values of CDH Family Members in Lung Adenocarcinoma" was retracted in 2023. Reasons: signs of a paper mill; suspected computer-generated content; unreliable results or conclusions; concerns about the data.

## 2. Materials and Methods

### 2.1. Patient Datasets

The expressing data of mRNAs (535 samples and 59 nontumor specimens) and clinical data were downloaded from TCGA database (https://cancergenome.nih.gov). The following samples were excluded: (1) the value of gene expression is “0” and (2) there is lack of survival data. 500 patients with LUAD with the corresponding clinical information were collected for our assays. DNA methylation profiles (Illumina HumanMethylation 450K) were downloaded from the GDC Tool.

### 2.2. Differentially Expressed Gene Analysis

The dysregulated genes were identified by the use of EdgeR (version 3.8) package in R software with FDR < 0.05 (adjusted *P* value) [14]. The heat map was constructed by the gplots package.

### 2.3. Survival Analysis

The Kaplan-Meier methods were applied to analyze the associations between the levels of CDH family members and the outcome of LUAD patients. Based on the expressing values of the autoselected best cutoff, all patients were divided in two groups (low and high). The Kaplan-Meier curves were plotted, and the log-rank tests were done to investigate the progression-free survival (PFS) and overall survival (OS) in LUAD. A *P* value < 0.05 is considered statistically significant.

The article "Expression Profile and Prognostic Values of CDH Family Members in Lung Adenocarcinoma" was retracted in 2023. Reasons: signs of a paper mill; suspected computer-generated content; unreliable results or conclusions; concerns about the data.

### 2.4. Associations between the Expression of mRNAs and Methylation of the CDH Family in LUAD

The correlation of the expression of CDH family members with the methylation of CpG sites in different regions of CDH family members was investigated using Pearson's correlation tests. We considered a *P* < 0.05 as statistically significant.

### 2.5. Gene Set Enrichment Analysis (GSEA)

For the exploration of biological signaling pathways involved in the expression of CDH members, GSEA was carried out in the high-expression and the low-expression groups based on the median expression of CDH members. The top five terms of KEGG were displayed. KEGG pathways with distinct enrichment results were confirmed based on the gene ratio and *P* value. FDR *q* < 0.05 was considered to be enrichment distinct.

### 2.6. Statistical Analysis

R 3.6.1 software and web resources were applied to carry out all statistical assays. *P* < 0.05 was considered indicative of statistical significance.

## 3. Results

### 3.1. Expressing Status of CDH Members in LUAD Specimens

To delve into the expressing pattern of CDH members in LUAD specimens, we analyzed their levels in 500 LUAD specimens and 59 nontumor lung specimens. Then, we calculated Pearson's correlation of CDH family genes, which was further applied to examine the possible associations in each member by the use of the corrplot package. As exhibited in Figure 1, the CDH family members were associated with a distinct degree. Then, the dysregulated CDH members were investigated applying the limma package and exhibited by the use of the pheatmap package (Figure 2(a)). In addition, we observed that the expression levels of CDH1 (Figure 2(b)), CDH2 (Figure 2(c)), CDH3 (Figure 2(d)), CDH4 (Figure 2(e)), CDH8 (Figure 2(f)), CDH15 (Figure S1A), CDH16 (Figure S1B), CDH17 (Figure S1C), CDH18 (Figure S1D), CDH24 (Figure S1E), and CDH26 (Figure S1F) were distinctly increased in LUAD specimens compared with nontumor lung specimens. In addition, we observed that the expression levels of CDH5 (Figure 2(g)), CDH6 (Figure 2(h)), CDH10 (Figure 2(i)), CDH13 (Figure 2(j)), CDH23 (Figure S1G), CDH19 (Figure S1H), and CDH22 (Figure S1I) were distinctly decreased in LUAD specimens. The detailed information was shown in Table 1.

### 3.2. The Associations of CDH Expression and Methylation in LUAD

It has been known that methylation is one of the most important mechanisms involved in the regulation of various genes, including tumor-related genes [15]. Pearson's correlation results showed that most CDH family members were negatively associated with the methylation level, such as CDH1 (Figure 3(a)), CDH2 (Figure 3(b)), CDH3 (Figure 3(c)), CDH4 (Figure 3(d)), and other CDH genes (Figure S2 and Figure S3). Our findings suggested the negative associations between expression and methylation levels of CDH members in LUAD.

The article "Expression Profile and Prognostic Values of CDH Family Members in Lung Adenocarcinoma" was retracted in 2023. Reasons: signs of a paper mill; suspected computer-generated content; unreliable results or conclusions; concerns about the data.

### 3.3. Identification of Survival-Related CDH Family Members in LUAD

To screen survival-related CDH family members, we performed Kaplan-Meier analysis in all LUAD patients based on the expression values of the autoselected best cutoff. We observed that 16 CDH family members were associated with the overall survival of LUAD patients, including CDH1 (Figure 4(a)), CDH2 (Figure 4(b)), CDH3 (Figure 4(c)), CDH4 (Figure 4(d)), CDH7 (Figure 4(e)), CDH8 (Figure 4(f)), CDH13 (Figure 4(g)), CDH15 (Figure 4(h)), CDH17 (Figure 4(i)), CDH18, CDH19, CDH20, CDH22, CDH23, CDH24, and CDH26 (Figure S4). In addition, 14 CDH family members were associated with progression-free survival of LUAD patients, including CDH2 (Figure 5(a)), CDH5 (Figure 5(b)), CDH7 (Figure 5(c)), CDH8 (Figure 5(d)), CDH1 (Figure 5(e)), CDH12 (Figure 5(f)), CDH15 (Figure 5(g)), CDH17 (Figure 5(h)), CDH18 (Figure 5(i)), CDH19, CDH20, CDH23, CDH4, and CDH26 (Figure S5). More importantly, we further performed multivariate analysis to determine the prognostic value of the above CDH family members and found that the expression levels of CDH17 (Figure 6(a)), CDH19 (Figure 6(b)), and CDH24 (Figure 6(c)) were independent prognostic biomarkers of the LUAD outcome.

### 3.4. GSEA Identifies CDH Member-Associated Pathways

To screen CDH member-associated pathways in LUAD, GSEA between CDH member high- and low-expression datasets was conducted to reveal distinct differences in the enrichment of MSigDB Collection. The results revealed that low expression levels of CDH17 were related to RNA_POLYMERASE and SPLICEOSOME (Figure 7(a)). Low expression levels of CDH19 were related to BASE_EXCISION_REPAIR, PROTEASOME, PYRIMIDINE_METABOLISM, RNA_POLYMERASE, and SPLICEOSOME (Figure 7(b)). High expression levels of CDH24 were related to CELL_CYCLE, HOMOLOGOUS_RECOMBINATION, NOTCH_SIGNALING_PATHWAY, PYRIMIDINE_METABOLISM, and SPLICEOSOME (Figure 7(c)).

## 4. Discussion

Alteration of biological markers in tumor tissues plays an important role in predicting the prognostic value of the LUAD patients [16, 17]. LUAD is a malignant disease which is very complex and heterogeneous in developments, progresses, and response to treatments [18]. To date, clinical biomarkers cannot display the whole prognostic significances for LUAD patients. Therefore, finding out novel prognostic biomarkers is very critical for LUAD patients.

With the development of high-throughput sequencing, it is possible for us to explore the expressing pattern of the gene family in various types of tumors and their clinical significance [19–21]. Our group examined the expressing patter and prognostic values of CDH members in LUAD. Previously, the dysregulation of CDH family members has been frequently reported. For instance, CDH5 expression was distinctly increased in gastric cancer and significantly associated with the recurrence [22]. Yang et al. reported that the levels of CDH13 were distinctly upregulated in breast cancer [23]. Importantly, CDH1, CDH2, and CDH12 were highly expressed in lung cancer [24–26]. However, the expression levels of the entire CDH members in LUAD have not been comprehensively studied. Here, we analyzed TCGA datasets and found that CDH1, CDH1, CDH3, CDH4, CDH15, CDH16, CDH17, and CDH24 were distinctly increased in LUAD tissues compared with nontumor specimens. In contrast, CDH5, CDH6, CDH8, CDH10, CDH13, CDH16, CDH18, CDH19, CDH22, CDH23, and CDH26 were distinctly decreased in LUAD specimens compared with nontumor specimens. These findings indicated that different CDH family members may play a different role in LUAD progression.

The article "Expression Profile and Prognostic Values of CDH Family Members in Lung Adenocarcinoma" was retracted in 2023. Reasons: signs of a paper mill; suspected computer-generated content; unreliable results or conclusions; concerns about the data.

Then, we analyzed the associations between the expression of CDH members and the methylation levels of cg sites in LUAD. Among the dysregulated CDH members (CDH1, CDH1, CDH3, CDH4, CDH15, CDH16, CDH17, CDH24, CDH5, CDH6, CDH8, CDH10, CDH13, CDH16, CDH18, CDH19, CDH22, CDH23, and CDH26), many CDH members, particularly for CDH1 and CDH26, were regulated by methylation levels. Our findings are in line with previous results for CDH1 [27].

To explore the prognostic value of CDH family members in LUAD, we performed Kaplan-Meier analysis and 15 survival-related CDH family members, including CDH1, CDH2, CDH7, CDH8, CDH4, CDH3, CDH15, CDH17, CDH24, CDH26, CDH13, CDH18, CDH19, CDH20, CDH22, and CDH23. To further determine the potential of the 15 survival-related CDH family members used as novel biomarkers for LUAD, we performed multivariate analysis and confirmed that CDH17, CDH19, and CDH24 were independent prognostic factors for LUAD patients. Previously, Jiang et al. reported that CDH17 expression was distinctly increased in gastric cancer and its silence suppressed the proliferation and metastasis of gastric cancer cells via regulating MMP2 [28]. CDH24 was reported to predict poor outcomes of gastric and colorectal cancers [29]. However, their function in LUAD has not been investigated. Further experiments are needed to further confirm our findings.

## 5. Conclusion

In summary, this study represented the expressing status of CDH members in LUAD and identified 18 differentially expressed CDH genes. CDH17, CDH19, and CDH24 were independent prognostic factors for LUAD patients. Our findings may inspire new clinical practices for patients with LUAD, including diagnosis, treatment, and prognosis.

The article "Expression Profile and Prognostic Values of CDH Family Members in Lung Adenocarcinoma" was retracted in 2023. Reasons: signs of a paper mill; suspected computer-generated content; unreliable results or conclusions; concerns about the data.

## Figures and Tables

**Figure 1:** Associations between CDH family members using the corrplot package.

**Figure 2:** The expressing pattern of CDH family members in LUAD. (a) The transcription levels of CDH genes in LUAD shown by the heat map. (b–j) The expression of CDH genes in LUAD and healthy control samples. ^∗^*P* < 0.05, ^∗∗^*P* < 0.01, and ^∗∗∗^*P* < 0.001.

**Figure 3:** Pearson's correlation between methylation levels and expression of (a) CDH1, (b) CDH2, (c) CDH3, and (d) CDH4.

**Figure 4:** (a–i) Kaplan-Meier analysis was used to explore the association between CDH family members and overall survival of LUAD patients.

**Figure 5:** (a–i) Kaplan-Meier analysis was used to explore the association between CDH family members and progress-free survival of LUAD patients.

**Figure 6:** Multivariate Cox regression analyses of clinicopathological features and CDH family members, including (a) CDH17, (b) CDH19, and (c) CDH24.

**Figure 7:** KEGG pathways associated with (a) CDH17, (b) CDH19, and (c) CDH24 based on a gene set enrichment analysis.

**Table 1:** The expressing pattern of CDH members in LUAD specimens and nontumor specimens based on TCGA datasets.

Gene	Normal	Tumor	LogFC	*P* value
CDH1	35.97208	78.74597	1.130329	3.24*E* − 21
CDH2	0.419067	1.682875	2.005675	0.01477
CDH3	2.824993	20.84318	2.883257	1.68*E*−20
CDH4	0.204208	0.381217	0.900574	0.003582
CDH5	41.97519	8.02393	−2.38716	2.88*E* − 34
CDH6	1.099119	0.703061	−0.64462	4.13*E* − 12
CDH7	0.008225	0.033671	2.033316	0.224584
CDH8	0.036871	0.060967	0.725548	0.039481
CDH9	0.005237	0.003907	−0.42267	0.618076
CDH10	0.148902	0.053452	−1.47803	1.78*E* – 10
CDH11	7.365005	9.212651	0.32293	0.792565
CDH12	0.016685	0.083754	2.327651	0.336363
CDH13	3.368875	1.045493	−1.68808	1.59*E* − 26
CDH15	0.226148	1.031876	2.189927	1.34*E* − 08
CDH16	0.153794	0.213401	0.472569	2.29*E* − 15
CDH17	0.088101	3.487431	5.306863	6.41*E* − 15
CDH18	0.006402	0.175256	4.774795	0.001259
CDH19	0.435657	0.090702	−2.26398	1.35*E* − 28
CDH20	0.052056	0.161722	1.63537	0.454749
CDH22	0.041982	0.025013	−0.74709	1.24*E* − 13
CDH23	0.711677	0.330682	−1.10578	4.98*E* − 20
CDH24	1.230606	3.896046	1.662641	2.77*E* − 19
CDH26	1.483066	1.820857	0.296035	0.001002

## Data Availability

The analyzed datasets generated during the study are available from the corresponding authors upon reasonable request.

## Supplementary Materials

Supplementary 1 Figure S1 (A-I): the expressing pattern of CDH family members in LUAD.

Supplementary 2 Figure S2: Pearson's correlation between methylation levels and expression of CDH family members, including CDH5, CDH6, CDH7, CDH8, CDH9, CDH10, CDH11, CDH12, and CDH13.

The article "Expression Profile and Prognostic Values of CDH Family Members in Lung Adenocarcinoma" was retracted in 2023. Reasons: signs of a paper mill; suspected computer-generated content; unreliable results or conclusions; concerns about the data.

Supplementary 3 Figure S3: Pearson's correlation between methylation levels and expression of CDH family members, including CDH24, CDH23, CDH22, CDH26, CDH15, CDH16, CDH17, CDH19, CDH18, and CDH20.

Supplementary 4 Figure S4: Kaplan-Meier assays were applied to explore the association between CDH family members and overall survival of LUAD patients.

Supplementary 5 Figure S5: Kaplan-Meier assays were applied to explore the association between CDH family members and progress-free survival of LUAD patients.

## References

[1] Hirsch F. R., Suda K., Wiens J., Bunn P. A. (2016). New and emerging targeted treatments in advanced non-small-cell lung cancer. *Lancet*.

[2] Cao M., Chen W. (2019). Epidemiology of lung cancer in China. *Thorac Cancer*.

[3] Balzer B. W. R., Loo C., Lewis C. R., Trahair T. N., Anazodo A. C. (2018). Adenocarcinoma of the lung in childhood and adolescence: a systematic review. *Journal of Thoracic Oncology*.

[4] Byers L. A., Rudin C. M. (2015). Small cell lung cancer: where do we go from here?. *Cancer*.

[5] Jacobsen M. M., Silverstein S. C., Quinn M. (2017). Timeliness of access to lung cancer diagnosis and treatment: a scoping literature review. *Lung Cancer*.

[6] Gheldof A., Berx G. (2013). Cadherins and epithelial-to-mesenchymal transition. *Progress in Molecular Biology and Translational Science*.

[7] Saito M., Tucker D. K., Kohlhorst D., Niessen C. M., Kowalczyk A. P. (2012). Classical and desmosomal cadherins at a glance. *Journal of Cell Science*.

[8] Yulis M., Kusters D. H. M., Nusrat A. (2018). Cadherins: cellular adhesive molecules serving as signalling mediators. *The Journal of Physiology*.

[9] Breier G., Grosser M., Rezaei M. (2014). Endothelial cadherins in cancer. *Cell and Tissue Research*.

[10] Pancho A., Aerts T., Mitsogiannis M. D., Seuntjens E. (2020). Protocadherins at the crossroad of signaling pathways. *Frontiers in Molecular Neuroscience*.

[11] Cardamone M. D., Bardella C., Gutierrez A. (2009). ERalpha as ligand-independent activator of CDH-1 regulates determination and maintenance of epithelial morphology in breast cancer cells. *Proceedings of the National Academy of Sciences of the United States of America*.

[12] Tang Q., Lu J., Zou C. (2018). CDH4 is a novel determinant of osteosarcoma tumorigenesis and metastasis. *Oncogene*.

[13] Zhao J., Li P., Feng H. (2013). Cadherin-12 contributes to tumorigenicity in colorectal cancer by promoting migration, invasion, adhersion and angiogenesis. *Journal of Translational Medicine*.

[14] Robinson M. D., McCarthy D. J., Smyth G. K. (2010). edgeR: a Bioconductor package for differential expression analysis of digital gene expression data. *Bioinformatics*.

The article "Expression Profile and Prognostic Values of CDH Family Members in Lung Adenocarcinoma" was retracted in 2023. Reasons: signs of a paper mill; suspected computer-generated content; unreliable results or conclusions; concerns about the data.

[15] Klutstein M., Nejman D., Greenfield R., Cedar H. (2016). DNA methylation in cancer and aging. *Cancer Research*.

[16] Villalobos P., Wistuba I. I. (2017). Lung Cancer Biomarkers. *Hematology/oncology clinics of North America*.

[17] Liu Z. J., Hou P. X., Wang X. X. (2021). An inflammation-related nine-gene signature to improve prognosis prediction of lung adenocarcinoma. *Disease Markers*.

[18] de Sousa V. M. L., Carvalho L. (2018). Heterogeneity in lung cancer. *Pathobiology*.

[19] Pareek C. S., Smoczynski R., Tretyn A. (2011). Sequencing technologies and genome sequencing. *Journal of Applied Genetics*.

[20] Tomczak K., Czerwińska P., Wiznerowicz M. (2015). The cancer genome atlas (TCGA): an immeasurable source of knowledge. *Contemporary oncology*.

[21] Zhang H., Ju Q., Ji J., Zhao Y. (2021). Pan-cancer analysis reveals FH as a potential prognostic and immunological biomarker in lung adenocarcinoma. *Disease Markers*.

[22] Inokuchi M., Higuchi K., Takagi Y. (2017). Cadherin 5 is a significant risk factor for hematogenous recurrence and a prognostic factor in locally advanced gastric cancer. *Anticancer Research*.

[23] Yang J., Niu H., Huang Y., Yang K. (2016). A systematic analysis of the relationship of CDH13 promoter methylation and breast cancer risk and prognosis. *PLoS One*.

[24] Ye T., Li J., Sun Z. (2020). Cdh1 functions as an oncogene by inducing self-renewal of lung cancer stem-like cells via oncogenic pathways. *International Journal of Biological Sciences*.

[25] Wang L., Peng Q., Sai B. (2020). Ligand-independent EphB1 signaling mediates TGF-*β*-activated CDH2 and promotes lung cancer cell invasion and migration. *Journal of Cancer*.

[26] Bankovic J., Stojsic J., Jovanovic D. (2010). Identification of genes associated with non-small-cell lung cancer promotion and progression. *Lung Cancer*.

[27] Liu G. (2018). CDH1 promoter methylation in patients with cervical carcinoma: a systematic meta-analysis with trial sequential analysis. *Future Oncology*.

[28] Jiang X. J., Lin J., Cai Q. H., Zhao J. F., Zhang H. J. (2019). CDH17 alters MMP-2 expression via canonical NF-*κ*B signalling in human gastric cancer. *Gene*.

[29] An C. H., Je E. M., Yoo N. J., Lee S. H. (2015). Frameshift mutations of cadherin genes DCHS2, CDH10 and CDH24 genes in gastric and colorectal cancers with high microsatellite instability. *Pathology Oncology Research*.

